The article "A Comparison between Accurate Unilateral Puncture Paths Planned by Preoperative and Conventional Unilateral Puncture Techniques in Percutaneous Vertebroplasty" was published in 2022. Journal: Comput Math Methods Med.

# A Comparison between Accurate Unilateral Puncture Paths Planned by Preoperative and Conventional Unilateral Puncture Techniques in Percutaneous Vertebroplasty

**DOI:** 10.1155/2022/6762530

**Published:** 2022-07-04

**Authors:** Yanchun Xie, Hongwen Gu, Wei Yongcun, Yuhui Zhao, Liangbi Xiang, Di Meng, Anna Wang, Hailong Yu

**Affiliations:** ^1^Department of Spine, General Hospital of Northern Theater Command, China; ^2^Panjin Liaoyou Gem Flower Hospital, China; ^3^Jinzhou Medical University, Jinzhou, China; ^4^Liaoning Dianli Central Hospital, China

## Abstract

**Objective:**

Comparison of the clinical and radiological effects of precise unilateral puncture pathway prepared by preoperative CT data and traditional unilateral puncture pathway in PVP administration for the treatment of osteoporotic vertebral compression fractures. *Summary of background data.* PVP is a commonly used vertebral augmentation operation for the treatment of painful spinal compression fractures. A percutaneous unilateral approach is routinely used to get access to the vertebral body. PVP has had positive clinical results in a number of prior investigations. Numerous difficulties and issues, including puncture difficulty, radiation exposure, cement leakage, spinal cord or nerve damage, and intraspinal hematoma, have been described in contrast.

**Methods:**

This prospective study included 300 patients with single-level lumbar osteoporotic vertebral compression fractures, 180 females and 120 males, with an average age of 71.5 years. PVP was performed on randomized subjects using two distinct puncture procedures. The patients were separated into two groups: Preoperative planning, in which a precise unilateral puncture path was established using preoperative CT data, and Conventional planning, in which multiple puncture procedures were used. The participants were followed up on after surgery and mostly assessed on clinical and radiological results. The visual analogue scale for pain and the 36-item Short Form Health Survey (SF-36) questionnaire for health status were used to assess clinical outcomes. Radiation dosage, bone cement distribution, vertebral body height, and kyphotic angle were used to evaluate radiological results.

**Results:**

Participants remained monitored for 12 to 28 months on average. 151 individuals were treated with accurate unilateral puncture paths planned by preoperative CT data percutaneous vertebroplasty and 149 patients were treated with conventional unilateral paths percutaneous vertebroplasty. The Preoperative planning group's operation time and radiation dose were significantly lower than the Conventional group's; nevertheless, the volume of injected cement was significantly higher in the Preoperative steering committee than in the Conventional group. All patients in both groups had much less pain after the operations when compared to their preoperative suffering. There were no statistically significant variations between groups when the visual analogue scale and the 36-Item Short Form Health Survey were compared. Neither group showed a substantial decrease in the kyphotic angle during the follow-ups. In the Preoperative planning group, the kyphotic angle improved much more than in the Conventional group. At 1 month postoperatively, 16 patients in the Conventional group experienced apparent discomfort in the puncture sites because to facet joint violation. At the latest follow-up, all of the patients' discomfort had vanished after receiving local block therapy.

The article "A Comparison between Accurate Unilateral Puncture Paths Planned by Preoperative and Conventional Unilateral Puncture Techniques in Percutaneous Vertebroplasty" was published in 2022. Journal: Comput Math Methods Med.

**Conclusion:**

Both preoperatively designed precise unilateral puncture pathways and traditional unilateral puncture procedures PVP are reasonably safe and effective for individuals with painful osteoporotic spinal compression fractures. Unilateral puncture courses planned via preoperative PVP, on the other hand, absorbed less radiation and operation time, as well as a good level of deformity correction and amount of injected cement, and caused less complications than traditional unilateral PVP.

## 1. Introduction

PVP is a minimally invasive, safe, and successful method for treating osteoporotic vertebral compression fractures (OVCF). PVP's pain alleviation rate in the treatment of OVCF has been reported to be as high as 90% [1–4]. PVP research nowadays focuses mostly on comparing the effects and consequences of unilateral versus bilateral penetration. Yilmaz [5] found that there was no significant difference between pain alleviation and vertebral height improvement between unilateral and bilateral puncture. However, unilateral puncture takes much less time, has less bone cement injection, and takes longer to puncture. Nevertheless, there is little information in the available literature on how to obtain unilateral exact puncture to produce a safe puncture path, sufficient bone cement dispersion, low bone cement leakage rate, good clinical effect, shorter operation times, and shorter fluoroscopy periods. If the puncture site is incorrect or the angle of inclination is insufficient, the anterior cortex of the vertebral body may be injured, resulting in bone cement leaking to the anterior side of the vertebral body and harm to the chest and abdominal cavity's essential organs. The upper endplate will be injured if the puncture point is too high or the puncture angle is excessively inclined to the cephalic side, resulting in bone cement leaking into the intervertebral space. The lower wall or lower endplate of the pedicle will be destroyed if the puncture point is too low or the tail angle is too great, leading in the leaking of bone cement through the lower endplate into the intervertebral space, and the puncture process will cause nerve root injury.

The article "A Comparison between Accurate Unilateral Puncture Paths Planned by Preoperative and Conventional Unilateral Puncture Techniques in Percutaneous Vertebroplasty" was published in 2022. Journal: Comput Math Methods Med.

The goal of this retrospective research was to use Preoperative planning to create an exact unilateral puncture path that would result in a safe, correct puncture, good clinical effect, bone cement diffusion filling, shorter operation time, and lower radiation exposure. The purpose of this prospective research was to compare preoperatively prepared proper unilateral puncture paths to traditional unilateral penetration using PVP in terms of clinical results, changes in the administered cement, and radiological results.

## 2. Materials and Methods

### 2.1. Patient Population

In this prospective study, 300 patients with single-level lumbar OVCF were treated with PVP from January 2012 to January 2015. There were 180 (60 percent) women and 120 (40 percent) men, with a mean age of 71.5 years (range: 55–91 years).

A nurse on the outpatient ward picked one of two distinct notes indicating one of two different puncture procedures after the patient had granted consent. One senior orthopedist specializing in spinal surgery conducted all of the surgeries. Each type of puncture procedure was performed alone by one surgeon at the Northern Theater General Hospital. As a result, the Conventional group had 149 patients and the Preoperative planning group had 151 patients. Northern Theater General Hospital's Institutional Review Boards & Ethics Committees both approved the study protocol. After a thorough explanation of the therapeutic procedure, all patients gave their informed consent prior to surgery.

#### 2.1.1. Inclusion Criteria

(1) A collapse of 15% or more of the vertebral height; (2) significant back pain due to a single-level OVCF that has been resistant to analgesic medicine for at least 2 weeks; (3) pain higher than 5 on a visual analogue scale, with tapping discomfort at the spinal process of the fractured vertebral body; (4) T1-weighted images with hypointense signal and T2-weighted images with hyperintense signal; and (5) bone asymmetry

#### 2.1.2. Exclusion Criteria

(1) Secondary osteoporosis (corticosteroids, endocrine disorders, and an inflammatory process); (2) inability to provide informed consent; (3) inappropriate coagulopathy; (4) overall physical state; (5) painless OVCF; (6) spinal metastatic cancer; and (7) neurological difficulties

### 2.2. Surgical Techniques

PVP operations were all done in the operating room, with the possibility of urgent decompression surgery. The patient was prone, with two transverse bolsters beneath his chest and pelvis. Then, to achieve relative reduction, we administered a mild 3-point reduction force to the broken vertebrae. Local anesthetic was employed in all operations to determine the patient's neurological condition. The C-arm was modified such that the damaged vertebral body had no bilateral shadow and the pedicles were symmetrical, with the same distance to the spinous process.

The article "A Comparison between Accurate Unilateral Puncture Paths Planned by Preoperative and Conventional Unilateral Puncture Techniques in Percutaneous Vertebroplasty" was published in 2022. Journal: Comput Math Methods Med.

Under fluoroscopy, the trocars were introduced through the lateral edge of the pedicle at 3 o'clock on the right side and 9 o'clock on the left side in the Conventional puncture group. When the needle tip approached the inner border of the pedicle under anteroposterior fluoroscopy, it showed that the trocars did not penetrate the vertebral canal situated in the vertebral body. Under lateral fluoroscopy, the trocars' tip was placed at the posterior margin of the vertebral body, and the trocars did not breach the canal.

In Preoperative planning group, all patients were placed in body surface locator on fracture vertebral body surface, and CT scan fracture vertebral body and surface locator was carried out to achieve the purpose of skin data visualization (Figure 1). CT data was imported into Minics software to carry out fracture vertebral body reconstruction and puncture path planning. In this study, there were three key points consisted of skin puncture point (Point A), vertebral bone puncture point (Point B), and intravertebral landing point (Point C) to complete the accurate unilateral puncture path (line). The lateral anterior cortex of the vertebral body intersected with the inner border of the contralateral pedicle at Point C. The tangent intersection of the central line of the transverse process and the lateral border of the pedicle, which had been horizontally translated a distance of a pedicle projection from its initial location, was designated as Point B. Point A was the intersection of the reverse extension line connecting Point C and Point B and the skin. The position of Point A can be determined by the body surface locator installed before the operation (Figure 2). According to the skin puncture point (Point A) planned before operation, puncture can be carried out without fluoroscopy (Figure 3(a)). Under fluoroscopy, vertebral bone puncture point (Point B) of the vertebral body can be found (Figure 3(b)). It signifies that the puncture path was safe if the point of the trocars was positioned at the inner edge of the pedicle under anteroposterior fluoroscopy and at the posterior margin of the vertebral body under lateral fluoroscopy. After that, the guide wire was inserted through the trocars channel into the vertebral body until the tip of the guide wire reached the anterior border of the vertebral body under lateral fluoroscopy and the inner margin of the contralateral pedicle under anteroposterior fluoroscopy. The guide wire's tip corresponded to Point C, which had been preoperatively determined (Figure 4). The timing of the surgery, the injection of bone cement, the radiation dosage, and the leaking of bone cement were all documented and compared (Figure 5). After 24 hours, all patients were released and told to avoid intense physical exertion for the next two months. At 1, 3, 6, and 12 months after the treatment, patients had follow-up consultations. Clinical and radiological evaluations were conducted prior to surgery as part of these follow-ups.

The article "A Comparison between Accurate Unilateral Puncture Paths Planned by Preoperative and Conventional Unilateral Puncture Techniques in Percutaneous Vertebroplasty" was published in 2022. Journal: Comput Math Methods Med.

### 2.3. Outcome Measures

Two spinal scale questionnaires were used to assess our patients' functional recovery. A VAS scale ranging from 0 (no pain at the base) to 10 (extremely severe pain) was used to quantify the overall discomfort (maximal imaginable pain at the summit). The patients' health was assessed using the 36-item Short Form Survey (SF-36) questionnaire. The form's Chinese counterpart has already gone through translation and validation testing. The surveys were completed preoperatively, as well as 1 month, 6 months, and 12 months after the operation.

Anteroposterior and lateral standing radiographs were collected to evaluate the vertebral height and kyphotic angle of the vertebral body in all patients before the surgery, at the time of discharge, and at 6 and 12 months after surgery. To use this scale, the program calculated the anterior height (AH) index and PH index of the broken vertebra on the same radiograph. The kyphotic angle was calculated by measuring the angle between the superior endplate at one level above the damaged vertebrae and the inferior endplate place at a single level underneath the fractured vertebrae.

### 2.4. Statistical Analysis

SPSS software, version 12 was used to conduct all statistical analyses (SPSS Inc., Chicago, IL). The 2 and Fisher exact tests were used to compare categorical variables. They are expressed as percentages and figures. Independent 2-sample *t* tests were used to obtain the mean and standard deviation of baseline continuous variables. Using paired *t* tests, the preoperative and postoperative ratings in each group were compared. *P* < 0.05 was considered statistical significance.

## 3. Results

Trocar penetration into the damaged vertebral body was performed correctly in all cases under C-arm supervision, and there were no intraoperative deaths in this research. The average length of time between follow-ups was 16.8 months (range: 12-28 months). After 12 months, 24 patients from both groups were missed during follow-ups and were eventually deleted. There were 5 deaths that were unconnected to the operations, and the other 19 instances were unable to be reached for further examination due to address or phone number changes. In the end, 276 people were included in the trial. 134 patients were treated with the traditional unilateral puncture procedure, while 142 patients were treated using preoperatively designed correct unilateral puncture pathways. The Conventional group had an 89.9% (134/149) follow-up rate, whereas the Preoperative planning group had a 94.0 percent (142/151) follow-up rate. In terms of patient demographic data, there have been no major variations among two categories (Table 1).

The article "A Comparison between Accurate Unilateral Puncture Paths Planned by Preoperative and Conventional Unilateral Puncture Techniques in Percutaneous Vertebroplasty" was published in 2022. Journal: Comput Math Methods Med.

In the Conventional and Preoperative planning groups, the mean volume of injected cement was 3.4 0.7 mL and 5.9 0.9 mL, respectively (*P* 0.01). The right unilateral puncture method (31.2 4.1 min) consumed substantially less time than the usual treatment (45.2 5.1 min) (*P* 0.01). The mean radiation dosage to each patient using the precise unilateral approach was 0.88 1.20 mSv, compared to 1.91 1.10 mSv in the other group, a statistically significant difference (*P* 0.01). Despite a lower dosage (0.14 0.20 mSv) in the correct unilateral approach compared to the traditional method (0.23 0.70 mSv), there was no significant difference in the mean radiation dose to the operator between the two groups (Table 1).

### 3.1. Clinical Results

Figure 3 depicts a graph of the VAS pain score. When compared to the preoperative period, both groups of patients experienced much less discomfort following the surgeries. The Preoperative planning group's mean pain score decreased from 8.1 1.4 before surgery to 3.7 1.1 at one month postoperatively (*P* < 0.01) and 2.6 1.3 at 12 months (*P* < 0.01). Similarly, the Conventional group's mean pain score dropped from 7.9 1.3 preoperatively to 4.0 1.2 at 1 month (*P* < 0.01) and 2.9 1.4 after 12 months (*P* < 0.01). There were no statistically significant differences between the groups when mean pain scores were compared at all time points, from preoperative through postoperative to final follow-up (Figure 6).

According to the well-being of the SF-36, physical functioning, role constraints due to physical health, bodily pain, general health perceptions, vitality, social functioning, role limitations owing to emotional issues, and general mental health are measured and summarized in Table 2. At each evaluation, there were no significant group differences in terms of SF-36 (*P* > 0.05).

The two groups' preoperative and postoperative radiographic evaluations are measured and summarized in Table 3. In the Conventional group, the average AH rose from 50.46% 11.28% percent preoperatively to 79.37 12.4% at 12 months postoperatively (*P* 0.01), and the PH altered from 81.57 11.6 percent to 89.63 11.13 percent (*P* > 0.05). The mean AH climbed from 51.13% 11.28% percent preoperatively to 74.24 12.36 percent at 12 months postoperatively (*P* 0.01), and the PH altered from 83.52 10.69 percent to 87.53 11.21 percent (*P* > 0.05) when compared to the Conventional group. The AH and PH were not significantly different in either group immediately after surgery or at the 12-month follow-up (*P* > 0.05). Furthermore, during follow-ups, both groups demonstrated a substantial decrease in kyphotic angle. The Preoperative planning group's kyphotic angle improved considerably from 18.73 8.22° before surgery to 9.65 5.11° at the 12-month follow-up, whereas the Conventional group's kyphotic angle fell dramatically from 17.88 7.18° preoperatively to 12.39 5.36° at the 12-month follow-up. The Preoperative planning group had a much higher decrease in the kyphotic angle than the Conventional planning group (*P* > 0.01).

The article "A Comparison between Accurate Unilateral Puncture Paths Planned by Preoperative and Conventional Unilateral Puncture Techniques in Percutaneous Vertebroplasty" was published in 2022. Journal: Comput Math Methods Med.

### 3.2. Complications

This research found no procedure-related complications. Extra-vertebral cement leakages were found in 12 of 158 patients (7.6%) treated with Preoperative planning and 22 of 151 patients (14.6%) treated with traditional approach (*P* 0.01). The neighboring intervertebral disc in 14 cases (4 in the Preoperative planning group and 10 in the Conventional group), the paravertebral soft tissue or vein in 11 cases (7 in the Preoperative planning group and 4 in the Conventional group), and the spinal canal in 9 cases were the sites of leakage (1 case in the Preoperative planning group and 8 cases in the Conventional group). During the follow-up period, 30 patients (9.7%) in 34 levels (including 15 patients (9.5%) in 16 levels in the Preoperative planning group and 15 patients (9.9%) in 18 levels in the Conventional group) encountered a new fracture. Four levels in the Preoperative planning group and five levels in the Conventional group had new broken vertebrae that were close to previously treated vertebrae. Eight patients with additional fractures required a second surgery (5 were treated using the Preoperative planning approach and 3 were treated using the Conventional technique), while the others were managed conservatively. At 1 month postoperatively, 16 patients (10.5 percent, 16/151) in the Conventional group showed apparent discomfort (VAS>5) at the puncture sites, which was caused by facet joint violation. At the latest follow-up, all of the patients' pain has vanished thanks to local block therapy.

The article "A Comparison between Accurate Unilateral Puncture Paths Planned by Preoperative and Conventional Unilateral Puncture Techniques in Percutaneous Vertebroplasty" was published in 2022. Journal: Comput Math Methods Med.

### 3.3. Key Points

Puncture difficulties, cement leakage, intraspinal hematoma, and nearby vertebral fracture have all been recorded as complications of unilateral PVP.

The goal of this study is to evaluate the clinical and radiological effects of PVP in the treatment of OVCF using precise puncture pathways designed using preoperative CT data.

PVP with precise puncture pathways designed using preoperative CT data received less radiation and took less time to perform, had a better degree of deformity repair, and had fewer complications than traditional bilateral PVP.

## 4. Discussion

The optimal treatment for vertebral body fractures should produce a rapid and long-term reduction in symptoms, as well as a long-term restoration of the kyphotic deformity created by the fracture. Vertebroplasty and kyphoplasty are minimally invasive percutaneous treatments that have been shown to enhance quality of life while also reducing pain. In a survey reported by Muijs SP6, good to very good clinical outcomes for vertebroplasty and kyphoplasty were identified, with substantial pain reduction postoperatively compared to preoperatively [6]. Both bilateral and unilateral PKP are reasonably safe and effective therapy for persons with painful osteoporotic spinal compression fractures, according to Yan2. Unilateral PKP, on the other hand, had a lower radiation dosage and operation duration, as well as a higher degree of deformity repair and fewer problems than bilateral PKP. The above research, we think, followed the idea of unilateral puncture sites, which needed a larger extraversion angle and lateral to the lateral edge of the pedicles. However, how to determine the distance of 5 mm to the lateral edge of pedicle and the extraversion angle under fluoroscopy is still a difficult problem in clinical practice. In addition, repeatedly fluoroscopy was still needed when skin puncture point and bone puncture point location were determined. Moreover, fully dispersed bone cement was required in the vertebral body, as well as minimum times of fluoroscopy was required for the puncture under unilateral puncture.

In this study, 3D CT data of fracture vertebral body were imported into mimic software to plan the key puncture points and puncture paths. To begin, Point C was found at the junction of the extension line of the contralateral pedicle and the quadrate cortex of the lateral curvature of the vertebral body, which was situated under the plane at the midpoint of the line between the upper and lower end plates. The following are the reasons behind the study's placement of Point C: First and foremost, the pedicle route can reach this location without causing injury to the spinal cord or nerve roots. Second, intraoperative fluoroscopy signs are visible, and bone cement was distributed more evenly over the whole vertebral body. Yan et al. found that unilateral puncture injected 3.4 mL of bone cement into each vertebral body while bilateral puncture injected 5.5 mL. The volume of bone cement injected into each section in this investigation was 6 ml, which was much more than that described in the literature. The increased amount of bone cement injection in this trial was due to the preoperatively designed puncture method, which was more favorable to complete dispersion of bone cement in the vertebral body, as well as the bigger volume of the lumbar vertebral body. The osteo-puncture site (Point B) in this investigation was found at the junction of the transverse process' midline and the lateral border of a pedicle that had been translated one pedicle distance horizontally outwards. The following factors were considered while establishing the location of Point B: First, this site ensures that the puncture path has a wider inclination angle than the typical entrance point. Second, the line between this Point B and Point C went through the pedicle of vertebral without harming the spinal canal. Finally, the fluoroscopy anatomic mark in the anterior-posterior location was more visible. On the basis of determining the position of Point B, the point of intersection between the extension line and the preoperative surface locator was the puncture point (Point A). According to the above-mentioned Preoperative planning method, fluoroscopy was not required when choosing the skin insertion place (Point A) during the procedure; X-ray fluoroscopy was only required when identifying Point B with evident anatomical signals. As a consequence, the findings of this study imply that the puncture time and fluoroscopy radiation dosage required were much lower than in the unplanned group.

The article "A Comparison between Accurate Unilateral Puncture Paths Planned by Preoperative and Conventional Unilateral Puncture Techniques in Percutaneous Vertebroplasty" was published in 2022. Journal: Comput Math Methods Med.

The incidence of bone cement leakage is currently not consistent throughout the literature, with the lowest being less than 5% and the largest being more than 80%. Although the majority of patients have no visible clinical signs, certain significant individuals may have neurological impairment, pulmonary embolism, and even death. Some studies found that operation technology influenced the rate of bone cement leakage to some extent, but most studies do not consider operation technology as an independent risk factor for bone cement leakage. However, improving operation technology can reduce the rate of bone cement leakage to some extent [7–21]. Three occurrences of significant clinical consequences caused by puncture mistakes were documented in the research by Schmidt R et al. [7]. Among them, 2 cases of bone cement seepage in spinal canal were caused by puncture needle penetrating the inner wall of pedicle, and 1 case of hematoma in spinal canal was caused by puncture errors during operation, which penetrated the inner wall of pedicle and dura mater, and damaged the small artery on the surface of spinal cord. Consequently, 2 patients underwent the second revision of the anterior approach again, and 1 patient died. It can be seen that the inaccurate puncture can cause serious clinical complications. In the PKP/PVP operation, whether unilateral or bilateral puncture was selected, the most concerned complications of clinicians were still leakage of bone cement. One of the most common causes of bone cement leaking in clinical practice was iatrogenic damage to the vertebral cortex induced by an incorrect puncture route. The medial cortex of the pedicle or the posterior cortex of the vertebral body will be injured if the puncture site is partial or the angle is too great, resulting in bone cement leaking into the vertebral canal.

To summarize, the first aspect to consider in the design of the puncture route and important puncture spots before the surgery was whether the puncture route would harm the pedicle and cortex of the vertebral body from the standpoint of horizontal anatomy. The line between the point of landing (Point C) in the vertebral body and the point of bone entry (Point B) in the vertebral body (the puncture path) in this study passed through the transverse process, the lateral wall of the pedicle, the pedicle, and the vertebral body, and then met the junction point between the extension line of the opposite pedicle and the anterior cortex of the vertebral body. The puncture path designed by this study can not only ensure the full dispersion of bone cement but also ensure that the puncture process will not damage the pedicle and vertebral cortex and will not cause iatrogenic injury and iatrogenic leakage of bone cement. Once the puncture path is close to the upper endplate, it can cause medical injury leakage of the upper endplate. According to the analysis of sagittal anatomy, the puncture path designed in this study reached the midpoint of the line between the upper and lower endplates of the vertebral body through the middle point of transverse process (Point B). To put it in another way, the distance between the puncture route and the upper and lower endplates was the same, which was a little difference compared to the typical puncture path close to the top endplates. The goal of decreasing the site of the puncture route in this study was not to harm the lower wall of the pedicle but rather to keep the puncture channel away from the upper endplate, reducing upper endplate cement leakage and increasing cement diffusion between the upper and lower endplates. This study has certain drawbacks. This prospective research may have a limited number of patients. Furthermore, the two groups had a shorter follow-up duration. To generalize our findings, more long-term follow-up investigations with a larger patient sample are needed.

The article "A Comparison between Accurate Unilateral Puncture Paths Planned by Preoperative and Conventional Unilateral Puncture Techniques in Percutaneous Vertebroplasty" was published in 2022. Journal: Comput Math Methods Med.

## 5. Conclusion

According to this study, PVP with both accurate unilateral puncture courses determined by preoperative CT data and conventional unilateral puncture pathways was a generally safe and effective treatment for those with painful OVCF. Both surgeries achieved satisfactory clinical results after a 12-month follow-up, but PVP with accurate unilateral puncture pathways needed less radiation and operation time, produced a better degree of deformity repair, and had fewer problems than PVP with traditional unilateral puncture paths. Long-term study will be required to assess the benefits of these relative features in the future.

## Figures and Tables

**Figure 1:** (a) Before the procedure, the body surface locator was put on the fracture vertebral body's body surface skin and secured appropriately. (b) Scanning the CT picture of the fractured vertebral body with the body surface locator. (c) A lumbar spine CT three-dimensional reconstruction picture using a body surface locator.

**Figure 2:** Before the procedure, use Mimics software to plan the puncture path and crucial puncture locations. (a) Point C was the intersection of the extension line of the inner edge of the contralateral pedicle and the anterior cortex of the vertebral body in the axial plane, Point B was the intersection of the midpoint of the transverse process and the lateral margin of the pedicle, which was horizontally translated one pedicle distance outwards, and Point A was the intersection of the extension line linked by Point C to Point B and the body surface locator. (b) Point C was the junction of the middle point of the line connecting the upper and lower endplates with the anterior cortex of the vertebral body in the sagittal plane. The intersection of the extension line linking Point C to Point B and the body surface locator may be used to identify (c) Point A.

**Figure 3:** (a) Point A may be identified without the use of an X-ray fluoroscopic by using a body surface finder. (b) The junction of the central line of the transverse process and the lateral edge of the pedicle, which was horizontally translated one pedicle distance outwards, was Point B under X-ray fluoroscopic.

The article "A Comparison between Accurate Unilateral Puncture Paths Planned by Preoperative and Conventional Unilateral Puncture Techniques in Percutaneous Vertebroplasty" was published in 2022. Journal: Comput Math Methods Med.

**Figure 4:** (a) The guide wire reaches the medial margin of the contralateral pedicle under anteroposterior fluoroscopy, and the tip of the guide wire was Point C. (b) The guide wire reached the front border of the vertebral body under lateral fluoroscopy, and the guide wire tip was in the center of the line between the upper and lower endplates.

**Figure 5:** Under anterior-posterior and lateral fluoroscopy, bone cement diffused fully in vertebral body.

**Figure 6:** Preoperative and postoperative mean VAS scores for the Conventional and Preoperative planning groups.

**Table 1:** Characteristics of the study population.

Characteristic	Conventional group	Preoperative planning group	*P*
Patients, no.	134	142	
Age, mean (yr)	71.5 ± 4.1	71.4 ± 3.6	0.06
Females, no. (%)	86(64.1)	89(62.7)	
BMD T score	−3.2 ± 0.8	−3.1 ± 0.7	0.19
Intraoperative measurement			
Operation time (min)	45.2 ± 5.1	31.2 ± 4.1	<0.01
Volume of the injected cement (mL)	3.4 ± 0.7	5.9 ± 0.9	<0.01
Radiation dose			
Patient	1.91 ± 1.10	0.88 ± 1.20	<0.01
Operator	0.23 ± 0.70	0.14 ± 0.20	<0.01

Unless otherwise stated, data is provided as mean + standard deviation.

BMD indicates bone mineral density.

**Table 2:** Comparison of the effects of the two techniques on 8 dimensions of SF-36 between patients.

Dimensions	Conventional group				Preoperative planning group			
	Preoperative	1mo	6mo	12mo	Preoperative	1mo	6mo	12mo
RF	33.6 ± 6.7	78.26 ± 11.2	78.46 ± 10.9	78.36 ± 11.4	34.16 ± 7.6	77.96 ± 10.7	78.16 ± 11.4	78.36 ± 11.2
RP	21.52 ± 12.0	74.6 ± 14.2	73..36 ± 8.9	74.61 ± 8.9	23.33 ± 14.51	77.22 ± 10.5	77.42 ± 9.8	74.23 ± 11.2
BP	28.76 ± 10.2	66,82 ± 9.4	68.46 ± 10.6	66.32 ± 9.9	31.47 ± 9.1	68.76 ± 10.9	70.88 ± 10.8	69.78 ± 9.9
GH	59.58 ± 8.0	74.22 ± 6.7	75.33 ± 5.4	74.24 ± 8.9	60.34 ± 9.7	74.19 ± 7.8	74.47 ± 8.9	74.47 ± 7.5
VT	51.61 ± 10.2	66.26 ± 8.8	69.18 ± 8.6	69.16 ± 7.6	52.35 ± 10.5	69.34 ± 11.0	68.76 ± 13.7	68.55 ± 15.9
SF	53.47 ± 12.7	69.48 ± 15.6	70.21 ± 17.3	70.19 ± 18.6	53.14 ± 11.0	70.78 ± 14.9	71.62 ± 140	71.32 ± 13.6
RE	58.68 ± 17.2	75.46 ± 13.5	74.78 ± 13.2	75.12 ± 14.3	58.12 ± 19.4	74.65 ± 16.3	75.56 ± 18.3	75.24 ± 17.5
MH	63.46 ± 11.0	74.36 ± 10.1	72.34 ± 9.2	73.67 ± 10.3	66.43 ± 11.2	74.67 ± 11.3	74.23 ± 10.3	74.23 ± 11.1

The mean and standard deviation are used to show the data. Physical functioning is denoted by PF; role limits are denoted by RP; bodily pain is denoted by BP; and general health perceptions are denoted by GH. VT stands for vitality. RE, role constraints due to emotional difficulties; SF, social functioning; MH stands for “general mental health”; 36-Item Short Form Health Survey (SF-36).

**Table 3:** The Conventional and Preoperative planning groups were assessed radiographically both before and after surgery.

	AH (%)			PH (%)			Kyphotic angle (°)		
	Preoperative	12mo	Improvement	Preoperative	12mo	Improvement	Preoperative	12mo	Improvement
Conventional group	51.13 ± 11.28	74.24 ± 12.36	23.11 ± 4.25∗†	83.52 ± 10.69	87.53 ± 11.21	4.01 ± 5.79	17.88 ± 7.18	12.39 ± 5.36	5.49 ± 3.36
Preoperative planning group	50.46 ± 11.28	79.37 ± 12.4	28.91 ± 5.43∗†	81.57 ± 11.6	89.63 ± 11.13	8.06 ± 3.57	18.73 ± 8.22	9.65 ± 5.11	9.08 ± 4.36†

∗Preoperative vs. 12-month follow-up, *P* < 0.05. † Conventional group vs. Preoperative planning group, *P* < 0.05. AH indicates anterior height; PH, posterior height.

The article "A Comparison between Accurate Unilateral Puncture Paths Planned by Preoperative and Conventional Unilateral Puncture Techniques in Percutaneous Vertebroplasty" was published in 2022. Journal: Comput Math Methods Med.

## Data Availability

The data used to support this study are available from the corresponding author upon request.
